The article "Relationship between feed efficiency indexes and thermography, blood, and ruminal parameters in pre-weaning dairy heifers" was published in 2020. Journal: PLoS One.

# Relationship between feed efficiency indexes and thermography, blood, and ruminal parameters in pre-weaning dairy heifers

**DOI:** 10.1371/journal.pone.0236118

**Published:** 2020-07-15

**Authors:** C. F. A. Lage, S. G. Coelho, H. C. Diniz Neto, V. M. R. Malacco, J. P. P. Rodrigues, J. P. Sacramento, V. A. Teixeira, F. S. Machado, L. G. R. Pereira, T. R. Tomich, M. M. Campos

**Affiliations:** 1 Department of Animal Science, School of Veterinary, Federal University of Minas Gerais, Belo Horizonte, Brazil; 2 Institute of Studies of the Humid Tropic, Federal University of South and Southeast of Pará, Xinguara, Pará, Brazil; 3 Department of Bioengineering, Federal University of São João Del Rey, São João del-Rei, Minas Gerais, Brazil; 4 Brazilian Agricultural Research Corporation (Empresa Brasileira de Pesquisa Agropecuária, EMBRAPA), National Center for Research on Dairy Cattle, Juiz de Fora, Brazil; University of Illinois, UNITED STATES

## Abstract

The objective of this study was to evaluate whether pre-weaning heifer calves divergent for residual feed intake (**RFI**) or residual feed intake and body weight gain (**RIG**) exhibit differences in thermography, blood, and ruminal parameters. Thirty-two Gyr heifer calves were enrolled in a 63-d trial and classified into 2 feed efficiency (**FE**) groups based on RFI and RIG (mean ± 0.5 SD). The groups were classified as high efficiency (**HE**) **RFI** (HE RFI, *n* = 9), **HE RIG** (HE RIG, *n* = 10), low efficiency (**LE**) RFI (LE RFI, *n* = 10), and **LE RIG** (LE RIG, *n* = 11). The amount of whole milk provided for each calf was calculated based on their metabolic weight at birth (42% x **BW**^**0.75**^). The liquid diet was divided into two meals at 0700 and 1400 h. The total solid diet (**TSD**) was composed of 92% concentrate and 8% of Tifton 85 hay chopped in 5-cm lengths, as fed. Intake was measured daily. Blood concentrations of insulin, beta hydroxybutyrate, urea, and glucose, and ruminal pH, N-NH_3_, and volatile fatty acids (**VFA**) were evaluated at 14, 28, 42, 56, and 70 days of age. Thermal images of the calves were taken with an infrared camera (FLIR T420, FLIR Systems Inc., Wilsonville, OR) on d 56 (±3) at 0600 h, before the morning feeding. Total VFA concentration and propionate as % of total VFA were 24.2% and 22.2% lower in HE RFI compared to LE RFI calves, respectively. On the other hand, acetate as % of total VFA was 10.6% greater in HE RFI than LE RFI calves. Blood urea concentration tended to be greater in LE RFI than HE RFI calves. High efficiency HE RIG tended to have 6.8% greater acetate and 15.4% lower propionate as % of total VFA than LE RIG. Blood insulin concentration was greater and blood glucose tended to be greater for LE RIG than HE RIG group. Low efficiency RIG group had greater left rib, left flank, and anus surface temperature measured by infrared thermography than the HE RIG group. Differences in ruminal fermentation do not seem to be associated with pre-weaning calves efficiency, while differences in protein metabolism seem to affect RFI during this phase. Infrared thermography appears to be correlated to RIG in pre-weaning heifer calves.

## Introduction

In milk production systems, feed corresponds to 50% of the total cost of production [1]; therefore, improving feed efficiency (**FE**) is essential to increasing profitability [2]. Feed efficiency indexes, as a tool to select more efficient animals, have been studied [3]. More specifically, residual feed intake (**RFI**) is a FE index calculated as the difference between actual and expected animal feed intake, at a certain level of production [4]. The independence of RFI from productive parameters led researchers to suggest that this measurement describes the inherent variation of basic metabolic processes, mainly related to intake and digestion, anabolism and catabolism, activity, and thermoregulation processes [5]. Understanding the physiological basis of divergence between high and low FE animals can help identify and select more efficient animals, while considering any negative impact it can have in physiological processes. In addition, development of potential physiological markers of feed efficiency can reduce the cost of identification and selection of efficient cows in future studies [6].

Some studies linked RFI during lactation with RFI during the growth phase, indicating that RFI may be a lifetime trait [7,8]. Understanding FE indexes during the growth phase can increase the progress in their use, assisting in animal selection decisions early in their productive life. However, most studies are executed during the post-weaning phase, and little is known about whether there is a relationship between FE in the pre-weaning phase and other phases of life in dairy cows.

The selection of slow-growing animals can be a problem associated with RFI [9]; thus, residual intake and body weight gain (**RIG**) was proposed as an alternative index to select efficiently growing animals. In a companion paper [10], we detailed feed efficiency measures and how the calves were ranked in terms of RFI and RIG indexes. In addition, we compared HE and LE groups for the 2 indexes, regarding performance body measurements, digestibility, energy partitioning, and nitrogen partitioning.

To our knowledge, no research has been conducted to evaluate the possible differences in ruminal and blood metabolites in groups divergent for FE indexes in pre-weaning dairy calves. Moreover, while research conducted by our investigative group concluded that thermography may have the potential to be used for screening phenotypical divergence in calves classified for residual body weight gain [11], no comparison of thermography parameters for the RIG index has been done. Therefore, the objective of this study was to evaluate whether pre-weaning heifer calves divergent for FE indexes exhibit differences in thermography, blood, and ruminal parameters.

## Material and methods

### Calves, housing, management, and treatments

This study was approved by the Ethics Committee of Embrapa Dairy Cattle (number: 7194210316). The study was conducted at the Farm of Embrapa Dairy Cattle, located in Coronel Pacheco, Minas Gerais, Brazil.

As stated above, the data presented in this paper is part of a study that classified calves into high and low feed efficiency groups using two feed efficiency indexes (RFI and RIG). A detailed description of methods, diets composition, performance data, calculation of indexes, and group classifications are provided in [10]. Briefly, thirty-two Gyr heifer calves (body weight at birth = 25.2 ± 3.2 kg) produced by in vitro fertilization and born during the autumn (April to June) were used. After birth, the calves were immediately separated from their dams, weighed, and had their umbilical cord immersed in iodine solution (10%). Colostrum was administered (10% of BW; >50g of IgG L) up to 6 h after birth. Blood samples were collected via jugular venipuncture up to 48 h post-birth to measure total plasma protein (g/dL) using an electronic refractometer (Palm Abbe PA203x, Misco, Cleveland, Ohio, USA). The calves were housed in a shed without lateral walls, in individual sand beds (1.25 x 1.75 m) contained by chains 1.2 m in length.

The amount of milk offered for each calf was 42% of their metabolic weight at birth. The mean weight of calves at birth was 25.2 ± 3.2 kg (mean ± SD). Consequently, the daily milk supply was 4.7 ± 0.46 L. Calves received transition milk until 3 days of age, and whole milk from the 4^th^ to the 77^th^ day of age divided into 2 equal meals offered at 0700 and 1400 h in nipple buckets (Milk Bar®, New Zealand). On the 78^th^ day of age, milk supply was reduced by half, and the heifer calves were weaned on the 81^st^ day of age. Water and total solid diet (**TSD**; hay and starter) were offered *ad libitum* in buckets (10% of refusals for solid diet). Milk samples were collected twice daily (morning and afternoon) and analyzed for total solids, crude protein, lactose, and fat. The solid diet was provided since the first day of life and composed of 92% starter (Soymax Rumen pre-initial, 18% flocculated, Total Alimentos, Três Corações, Minas Gerais, Brazil) and 8% Tifton 85 (*Cynodon* spp.) hay chopped in 5-cm lengths, as fed. Samples of the TSD were collected 3 times a week, and composited and homogenized weekly.

Individual refusals were collected daily and were composited weekly. Milk, TSD, and water intake were measured individually. Daily intakes of milk, TSD, and water were calculated by the difference between offers and refusals. Feed and water were weighed using a bench scale (9094 plus, Toledo®, São Bernardo do Campo, São Paulo, Brazil) and a portable scale (WH-A04, WeiHeng, China), respectively. Body weight was recorded before the morning meal on days 3 and 7 after birth, and weekly from day 8 onward.

Solid feed was offered since the first day of life, but feed efficiency evaluations started with 14 d of age since there was no expressive solid intake before this age. Intake and performance were evaluated from the 14^th^ to the 77^th^ day of age to calculate the indexes based on 63 days of observation [12]. The growth rate of the animals was modeled by linear regression of BW against time over the trial duration, and the regression coefficients were calculated for the average daily gain (**ADG**) of each animal. Mean daily feed intake was calculated for each animal over the trial period and corrected for DM. The average metabolic weight (BW^0.75^) was calculated using the BW at the 46th day of age, which was the middle of the test period.

Dry matter intake, BW^0.75^, and ADG were used to estimate RFI and residual body weight gain (**RG**) using linear regressions [4], where RFI and RG were calculated as the difference between actual and predicted DMI and ADG respectively, as follows:

$$Y_{j}=\beta_{0}+\beta_{1}\left(BW^{0.75}{}_{j}\right)+\beta_{2}\left(ADG_{j}\;or\;DMI_{j}\right)+e_{j},$$

where Yj is the standardized DMI (RFI) or ADG (RG) of calf j, β0 is the intercept, β1 is the regression coefficient for BW^0.75^, β2 is the regression coefficient for ADG (RFI) or DMI (RG), and ej is the error term for calf j. In the present study, RG was not used as an FE index. The RG calculation was performed to estimate RIG. To calculate RIG, the residues for RFI and RG were added as [9]:

RIG=[RFIx(‐1)]+RG

Based on these indexes, the animals were classified into four groups: high efficiency (**HE**) and low efficiency (**LE**) for RFI and RIG. HE indicated RFI < 0.5 SD below the mean (n = 9) and RIG > 0.5 SD above the mean (n = 10), while LE indicated RFI > 0.5 SD above the mean (n = 10) and RIG < 0.5 SD below the mean (n = 11). The remaining animals were classified as intermediate and were not included in subsequent analyses.

### Blood collection and analysis

To determine the concentration of beta hydroxybutyrate (**BHB**), urea, and glucose, blood samples were taken at 14, 28, 42, 56, and 70 days of age; to determine the concentration of insulin, blood samples were taken at 28, 42, 56, and 70 days of age. All blood samples were taken via venipuncture of the jugular vein, 3 h after the morning meal. Tubes without anticoagulant for insulin, BHB, and urea, and with fluoride EDTA for glucose (Vacutainer; Becton, Dickinson and Company) were used. The tubes were stored on ice until centrifugation at 1,800 × G for 10 min at room temperature (22–25°C).

Aliquots of serum and plasma were stored at −20°C until further analysis. Glucose and urea were measured using a colorimetric enzymatic method (Kovalent do Brasil Ltd., Rio de Janeiro, Brazil). Insulin was analyzed using a Bovine ELISA kit (Bovine Insulin ELISA, Kit No. 10-1201-01, Mercodia AB, Uppsala, Sweden). The coefficients of inter- and intra-assay variation were 11.2% and 9.1%, respectively. BHB determination was performed using an enzyme kinetic kit (RANBUT kit—Ref.: RB 1007; RANDOX Laboratories–Life Sciences Ltd., Crumlin, UK). All readings were performed on an EON microplate spectrophotometer (Biotek Instruments Inc., Winooski, Vermont, USA).

### Rumen variables and analysis

Ruminal fluid samples were collected at 14, 28, 42, 56, and 70 days of age using an esophageal tube, 3 h after morning feeding. The liquid was double filtered through cheesecloth, and pH was measured (Mettler Toledo®, Columbus, Ohio, USA).

For N-NH_3_ determination, 5 mL of filtered ruminal liquid was acidified with 1 mL of sulfuric acid (500 mL/L) and stored at −20°C until further analysis. Analyses were performed after distillation of Kjeldahl with magnesium oxide and calcium chloride according to method 920.03 [13]. For volatile fatty acid (**VFA**) determination, 1 mL of 20% metaphosphoric acid was added to 10 mL of filtered ruminal liquid and stored at −20°C. Samples were defrosted at room temperature (22–25°C) and centrifuged at 13,000 rpm for 10 minutes. The samples were analyzed by high performance liquid chromatography (Waters Alliance and 2695 Chromatograph, Waters Technologies of Brazil LTDA, Barueri, São Paulo, Brazil).

### Infrared thermography

Thermal images of the calves were taken with an infrared camera (FLIR T420, FLIR Systems Inc., Wilsonville, Oregon, USA) on day 56 (±3) at 0600 h, before the morning feeding. The standard distance between thermograph and the target anatomical region was 0.5-m. The FLIR T420 default settings values for emissivity (0.98) and reflectance temperature (20ºC) recommended for animal skin or watery surface (eye) were used [14]. All thermal images were obtained in a roofed area, in the same place where the animals were housed (sand beds in tie-stalls). Calves were manually restrained during the evaluations, with no manipulation of the evaluated areas. Markings were used to ensure 0.5 m of distance between the animal restrained and the photographer. The evaluated anatomical regions were eye, jaw, muzzle, left-side ribs, left-side flank, right front limb, anus, and vulva. The average ambient temperatures and relative humidity recorded during imaging evaluations ranged between 13.8ºC and 20.8°C and 89% and 99%, respectively. The generated images were processed and interpreted using the FLIR Tools 5.6 software (FLIR Systems Inc.).

To establish a constant area of evaluation, a figure was drawn on the image surface, and it was then dragged to the region of the skin located in the chosen area [15]. Only the maximum temperature within each delimited area was considered to reduce the interference of factors such as contamination by water, feces, urine, or contact with colder surfaces, which could influence the thermogram. The rectal temperature of each animal was measured immediately after the thermal image evaluations using a digital thermometer (TH198, GTech, Rio de Janeiro, Brazil).

### Statistical analyses

Statistical analysis was performed using SAS software (version 9.4, SAS Institute Inc., Cary, North Carolina, USA). To evaluate the effects of efficiency in the groups, the MIXED procedure was used, according to the model:

$$Y_{ijk}=\beta_{0}+\beta_{1}A_{ij}+\beta_{2}B_{ij}+G_{i}+M_{k}+{GM}_{ik}+\delta_{ij}+\varepsilon_{ijk}$$

where Y_ijk_ is the dependent variable, β_0_ is the intercept, β_1_A_ij_ is the regression coefficient for the covariate initial BW, β_2_B_ij_ is the regression coefficient for the covariate total serum protein, G_i_ is the fixed effect of efficiency group (RFI or RIG), M_k_ is the fixed effect of repeated measure (day or week), GM_ik_ is the fixed effect of interaction between group and repeated measure, δ_ij_ is the random error between animals within treatment, and ε_ijk_ is the random error between measurements within animals. The best covariance structure for repeated measures was chosen by the lower corrected Akaike information criteria (**AICc**). For significative interaction between group and repeated measure, the differences among groups within measures were evaluated using the SLICE statement. For thermography data, the effects of repeated measures and its interaction with treatment were not included in the model and one random error term was used. Significance of the effects was declared at *P* ≤ 0.05, and tendency was accepted when 0.05 ≤ *P* ≤ 0.10.

## Results

### Residual feed intake

Average RFI for the HE group was −0.052 kg/d, and for the LE group, it was 0.049 kg/d (SEM = 0.010, *P* < 0.01). The HE RFI consumed 8.9% less than the LE RFI group. Total intake was 0.76 and 0.84 kg/d for the HE and LE RFI groups, respectively (SEM = 0.02, *P* = 0.002). Average daily gain was 0.60 and 0.59 kg/d for the HE and LE RFI groups, respectively (SEM = 0.02, *P*-value = 0.67), and body weight was 48.2 and 46.6 for the HE and LE RFI groups, respectively (SEM = 0.77, *P* = 0.17) [10].

No statistical differences (*P* > 0.17) were observed for ruminal pH, N-NH_3_ concentration (%), and proportion of butyrate (%VFA) between HE and LE RFI groups (Table 1). Total VFA concentration (μmol/mL) in ruminal fluid was greater (*P* = 0.001) for LE than HE RFI group. In addition, propionate (%VFA) was greater in the LE RFI group (*P* = 0.002), while acetate (% VFA) was lower for this group (*P* = 0.01).

**Table 1:** Rumen parameters in pre-weaning calves (14 to 77 days old) classified as high efficiency (HE) and low efficiency (LE) for RFI and RIG.

Item	RFI^1^		SEM^5^	*P*-value^6^	RIG^2^		SEM^5^	*P*-value^6^
	HE^3^	LE^4^			HE	LE		
N-NH_3_, %	14.7	15.6	0.71	0.31	16.7	16.2	0.90	0.67
pH	6.52	6.31	0.109	0.17	6.39	6.36	0.089	0.79
Total VFA, μmol/mL	32.9^a^	43.4^b^	1.99	0.001	34.6	39.8	2.27	0.11
*VFA*, *% of total VFA*								
Acetate	0.75^a^	0.67^b^	0.020	0.01	0.74	0.69	0.019	0.08
Butyrate	0.04	0.06	0.008	0.14	0.05	0.05	0.006	0.75
Propionate	0.21^a^	0.27^b^	0.013	0.002	0.22	0.26	0.015	0.06

^a,b^Means with different letter superscripts differ at P ≤ 0.05.

^1^Residual feed intake.

^2^Residual intake and body weight gain

^3^High efficiency

^4^Low efficiency

^5^Standart error of the means

^6^Main effect of group; Treatment × week interactions were, *P* ≥ 0.10, except total VFA (μmol/mL) (*P* = 0.017), acetate (%VFA) (*P* = 0.034) and propionate (%VFA) (*P* = 0.015) for RFI groups and *P* ≥ 0.11 for all variables in RIG groups.

A significative treatment × week interaction was observed for total VFA concentration (*P* = 0.017). Low efficiency RFI group had greater ruminal VFA concentrations at 28 and 42 d of age in comparison to HE RFI group (Table 1; Fig 1). A significative treatment × week interaction was also observed for ruminal acetate and propionate concentration (%; *P* = 0.034 and *P* = 0.015, respectively). Acetate concentration was lower in the LE RFI group at 28 and 42 d of age, while propionate concentration was greater in the LE than in the HE RFI group at 28, 42, and 56 d of age (Table 1; Fig 1).

**Fig 1:** (A) VFA (μmol/mL), (B) acetate (% VFA) and propionate (% VFA) in ruminal fluid of heifer calves classified as high efficiency (HE) and low efficiency (LE) of residual feed intake (RFI) from the 3^rd^ to the 11^th^ week of age. *represents the existence of difference between treatments (*P* < 0.05) in the week. Error bars represent standard error of the mean (SEM).

Blood BHB, glucose, and insulin concentrations did not differ between RFI groups (*P* > 0.22) (Table 2). Blood urea concentration tended (*P* = 0.06) to be greater in LE than HE RFI group.

**Table 2:** Blood parameters in pre-weaning heifer calves (14 to 77 days old) classified as high efficiency (HE) and low efficiency (LE) for RFI and RIG.

Item	RFI^1^		SEM^5^	*P*-value^6^	RIG^2^		SEM^5^	*P*-value^6^
	HE^3^	LE^4^			HE	LE		
BHB, μg/L	0.51	0.58	0.038	0.22	0.53	0.57	0.037	0.52
Glucose, mg/dL	125	123	6.8	0.84	118	125	2.7	0.07
Insulin, pmol/L	2.50	2.75	0.185	0.34	2.47	3.31	0.230	0.01
Urea, mg/dL	18.4	21.4	1.02	0.06	19.6	21.2	0.74	0.12

^1^Residual feed intake

^2^Residual intake and gain

^3^High efficiency

^4^Low efficiency

^5^Standart error of the means

^6^Main effect of group; Treatment × week interactions were, *P* ≥ 0.21 for RFI groups and *P* ≥ 0.48, except blood insulin concentration (*P* = 0.001) for RIG groups.

Skin surface temperature measured by infrared temperature did not differ between RFI groups, but a moderate correlation (0.47, *P* = 0.048) between flank temperature and RFI was observed (Tables 3 and 4).

**Table 3:** Skin surface temperature measure by infrared thermography in pre-weaning heifer calves (56 days old) classified as high efficiency (HE) and low efficiency (LE) for RFI and RIG.

Item	RFI^1^		SEM^5^	*P*-value^6^	RIG^2^		SEM^5^	*P*-value^6^
	HE^3^	LE^4^			HE	LE		
Temperature (ºC)								
Anus	37.7	38.2	0.24	0.13	37.4	38.2	0.24	0.03
Left eye	36.2	36.2	0.35	0.99	35.9	36.3	0.24	0.32
Left flank	30.8	32.4	0.82	0.18	30.8	30.9	0.63	0.03
Left foot	26.4	24.5	1.19	0.28	25.3	24.2	1.11	0.50
Left jaw	32.6	33.1	0.39	0.43	31.6	32.7	0.53	0.17
Left rib	32.7	33.1	0.52	0.58	32.1	33.6	0.42	0.02
Muzzle	22.8	22.5	0.79	0.74	22.6	22.3	0.75	0.80
Rectal	38.3	38.3	0.14	0.89	38.3	38.4	0.15	0.15
Vulva	36.2	36.7	0.29	0.23	36.2	36.7	0.22	0.15

^1^Residual feed intake

^2^Residual intake and gain

^3^High efficiency

^4^Low efficiency

^5^Standart error of the means

^6^Main effect of group

**Table 4:** Correlations between feed efficiency indexes (RFI and RIG) and skin surface temperature.

Item	RFI^1^		RIG^2^	
	R^3^	*P*-value^4^	R	*P*-value
Anus temperature	0.33	0.17	-0.34	0.13
Eye temperature	0.11	0.67	-0.13	0.57
Flank temperature	0.47	0.05	-0.59	0.01
Foot temperature	-0.31	0.22	0.33	0.16
Jaw temperature	0.34	0.15	-0.27	0.23
Muzzle temperature	-0.05	0.84	0.13	0.57
Rectal temperature	0.01	0.97	-0.06	0.79
Rib temperature	0.30	0.22	-0.45	0.05
Vulva temperature	0.24	0.31	-0.18	0.42

^1^Residual feed intake

^2^Residual intake and gain

^3^Correlation coefficients

^4^Main effect of group

### Residual feed intake and body weight gain

The average RIG for the HE group was 0.080 kg/d, and for the LE group, it was −0.077 kg/d. The HE RIG group had an 8.6% greater ADG than the LE RIG group (Table 2). Total intake was 0.78 and 0.80 kg/d for the HE and LE RFI groups, respectively (SEM = 0.010, *P* = 0.08). Average daily gain was 0.60 and 0.55 kg/d for the HE and LE RFI groups, respectively (SEM = 0.02, *P*-value = 0.04), and body weight was 47.8 and 46.3 for the HE and LE RFI groups, respectively (SEM = 0.25, *P*-value < 0.001) [10].

No differences in ruminal parameters between the HE and LE RIG groups were observed (Table 1), except a tendency to greater ruminal proportion of acetate (%VFA) (*P* = 0.08) and a lower proportion of propionate (%VFA) (*P* = 0.06) concentrations in HE RIG compared to LE RIG group.

Blood insulin concentration was greater (*P* = 0.02) for LE than for HE RIG group (Table 2). Blood glucose concentration also tended (*P* = 0.06) to be greater in the LE RIG group compared to the HE RIG group, but no differences in BHB and urea between RIG groups were observed. In addition, a treatment × week interaction for blood insulin concentration was observed (*P* = 0.001). Insulin was greater in LE compared to HE RIG animals at 56 days of age (Fig 2).

**Fig 2:** Blood insulin (pmol/L) concentration from 28 to 70 days of age in animals classified as HE or LE RIG. Asterisk (*) represents the existence of difference between treatments (*P* < 0.05). Error bars represent standard error of the mean (SEM).

The LE RIG group had greater (*P* = 0.03) left rib, left flank, and anus surface temperature measured by infrared thermography compared to the HE RIG group (Table 3). Hence, moderate correlations between flank (−0.594, *P* = 0.005) and rib temperature (−0.446, *P* = 0.048) with RIG were observed.

## Discussion

The objective of the present study was to evaluate whether pre-weaning calves divergent for FE indexes (RFI and RIG) exhibit differences in thermography, blood, and ruminal parameters. Clear evidence of differences in these parameters when using RFI or RIG as indexes for calves was observed for proportions of acetate and propionate in rumen VFA, blood glucose, insulin and urea depending on the FE index evaluated. The results also indicated differences in body surface temperatures when the calves were classified based on RIG but not RFI. Results from the current study indicates divergences on physiological basis underlying RFI and RIG and opens the perspective for future studies on a better understanding of how these differences affect productive traits of lactating dairy animals. Complementary results on performance body measurements, digestibility, energy partitioning, and nitrogen partitioning were described by [10].

### Residual feed intake

Residual feed intake is defined as the difference between observed and expected feed intake based on the requirement to support both maintenance and growth [16]. High-efficiency RFI animals eat less than average to support certain levels of production [4], and in the present study, HE RFI calves had an 8.6% less DM intake than LE RFI calves [10].

No differences in pH and N-NH_3_ between RFI groups were observed. Other studies that also used esophageal tube did not find differences in ruminal pH between HE RFI and LE RFI [17,18], demonstrating the same rumen environment conditions between RFI groups.

In the present study, calves with greater solid intake (LE RFI group) also had greater total VFA (μmol/mL). Similar results were also observed in LE RFI animals under feedlot conditions fed a grain-based diet [17]. Since rumen molar concentration of VFA is determined by its rates of production and absorption, greater availability of fermentable substrate in rumen can result in greater ruminal molar concentrations of VFA [19]. In addition, LE RFI calves had greater ruminal propionate and lower acetate (as % of total VFA), which was also observed by [17]. These results may be related to the lower passage rate in HE RFI calves. Although passage rate was not measured in the present study, it is reported in the literature that lower intake can reduce passage rate and therefore, increase fiber degradability and acetate production [20,21].

Differences in ruminal fermentation do not seem to be associated with pre-weaning calves' efficiency. A possible reason why HE RFI group kept the same ADG eating less and with lower VFA concentration may be related to more efficient post-ruminal digestion and absorption of nutrients in that group. Data from the same study presented in companion paper already published [10], showed that HE RFI group had greater crude protein and ether extract total tract digestibility, and tended to have improved total DM and organic matter total tract digestibility [10]. Because of a non-developed rumen, pre-weaning calves are largely dependent on intestinal digestion for the absorption of nutrients, and that appears to be the factor responsible for the RFI difference between the groups in this current experiment.

Blood concentration of metabolites and hormones can be a useful tool to understand differences in metabolism. Several RFI studies have evaluated blood parameters to understand differences in feed efficiency and tried to detect potential physiological markers for FE [22,23]. In the present study, no differences in glucose, insulin, and BHB were observed. These results are in accordance with other studies performed in growing animals [6,24] even though some observed a tendency (*P* < 0.10) for greater insulin in the LE RFI groups [25] or a weak correlation between high insulin values and greater RFI values [6].

In young ruminants, the main contribution to the plasma concentration of butyrate is related to its production in the rumen [26]. Therefore, the similar ruminal butyrate concentration (% of total VFA) between RFI groups, may explain the lack of differences in blood BHB of pre-weaning calves in the current study.

Low-efficiency RFI group tended to have greater blood urea concentrations in comparison to the HE RFI group. An association between greater concentrations of blood urea and LE RFI has been previously reported in the literature [25,27]. This is often related to greater protein intake [6]; however, data from the same calves presented in the companion paper [10], demonstrated that the LE RFI group had greater protein intake but similar nitrogen retention [10]. Protein intake does not seem to be the main reason underlying differences in blood urea, which suggests protein metabolism as a possible key point that determines differences in FE in pre-weaning dairy calves. Urea is a product of protein degradation [28], and greater blood urea concentration in LE RFI heifers can be related to greater AA catabolism in less efficient animals. There is evidence that LE RFI animals are more susceptible to stress and that they are more prone to mobilize muscle from the tissue, which can contribute to the increase in blood urea concentration [27]. However, more studies are needed to better understand this mechanism in pre-weaning dairy heifers.

Previous studies reported correlations between heat production and skin surface temperature measured by infrared thermography [29,30]. Since heat production was reported to account for up to 73% of the variation in RFI [5], we hypothesized that more efficient pre-weaning calves would have a decrease in heat production, which could be demonstrated by lower skin surface temperature. However, this hypothesis was not confirmed in the present study since no differences in skin surface temperature were observed between the RFI groups. Moreover, data presented in the companion paper [10] showed no differences in heat production measured by respiration chamber between the RFI groups. In accordance with that, [11], did not observe differences in skin surface temperature between RFI groups, although finding greater heat production in HE RFI compared to LE RFI, measured by the face mask. Contrary to our findings, previous experiments reported greater skin surface temperature measured by infrared thermography in post-weaning LE RFI cattle [15,31]. Evaluations of thermography during the current study were executed in the animals’ own stalls in thermoneutral conditions for calves Gebremedhin. The little knowledge available in the literature regard the interrelationship between RFI and IR temperature for pre-weaning dairy calves is not consistent [11 and the present study], and more studies are needed, but our results showed the limitation of IR thermography technique to differentiate divergent animals for RFI.

### Residual feed intake and body weight gain

Residual feed intake and body weight gain were proposed to be an intermediary index between RFI and RG [9]. Hence, the observed differences in intake and performance between the groups in this trial met the purpose of the index. A detailed discussion about performance and intake can be found in the companion paper [10].

As discussed above for RFI, changes in VFA concentration and percentage of each VFA followed intake parameters. The tendency to greater availability of fermentable substrate in rumen appears to be responsible for the tendency of greater molar concentrations of VFA in LE RIG compared to HE RIG group. In addition, the tendency to greater ruminal propionate (% of total VFA) and acetate (% of total VFA) proportion in LE RIG compared to HE RIG may be related to differences in passage rate between the groups.

The LE RIG group had greater blood insulin concentration at 56 d of age and tended to have greater glucose concentration. The secretion of insulin depends on the rate of nutrient absorption in the small intestine, feed composition, and neuroendocrine signaling to the pancreas [32]. Low-efficiency RIG animals tended to have greater DM intake, which could affect the appearance of nutrients, including glucose in the blood. Greater blood glucose would in turn stimulate the secretion of insulin, increasing the plasma concentration of this hormone [32]. However, the difference in insulin between the groups at 56 d of age is difficult to explain, since no differences in management between the groups happened at 56 d of age, and no important differences in blood glucose at 56 d of age between the groups were observed.

As mentioned before, one of our hypotheses was that HE RIG animals would dissipate less heat through the skin, reflecting lower heat production due to a possible more efficient metabolism. Although LE RIG animals had a greater left rib, left flank, and anus surface temperatures compared to HE RIG measured by infrared thermography, no differences in heat production measured by respiration chamber, presented in the companion paper [10], between RIG groups were observed.

These results do not corroborate with our initial hypothesis that skin surface temperature would reflect differences in heat production between HE and LE RFI groups; however, moderate correlations between surface temperature in some regions and RIG were observed. It is not clear which mechanism links greater efficiency and lower skin surface in RIG groups. Thus, more research is needed to investigate the relationship between RIG and skin surface temperature measured by thermography.

### Final considerations

Total ruminal VFA concentration and the proportions of acetate and propionate (% of total VFA) were greater in the LE RFI and RFI groups. Therefore, ruminal fermentation does not seem to be associated with pre-weaning heifer calves FE. Blood urea concentration was greater in the LE RFI group, suggesting protein metabolism as a possible key point determining differences in FE in pre-weaning dairy calves. Infrared thermography seems to be correlated to RIG but not to RFI; however, the mechanism linking skin surface temperature to RIG is not clear. This study indicates differences in physiological basis underlying RFI and RIG; therefore, more research needs to be conducted to better understand how these differences can affect the productivity of lactating cows and which index has better potential to improve the selection of more efficient animals.

## Supporting information

S1 Database (XLSX)
